This article has been retracted.

# A Deep Learning Filter that Blocks Phishing Campaigns Using Intelligent English Text Recognition Methods

**DOI:** 10.1155/2022/5036026

**Published:** 2022-05-30

**Authors:** Yonghui Tang, Fei Wu

**Affiliations:** ^1^Shaoyang University, Shaoyang 422000, China; ^2^Hunan Institute of Engineering, Xiangtan 411101, China

## Abstract

Most of the sophisticated attacks in the modern age of cybercrime are based, among other things, on specialized phishing campaigns. A challenge in identifying phishing campaigns is defining a classification of patterns that can be generalized and used in different areas and campaigns of a different nature. Although efforts have been made to establish a general labeling scheme in their classification, there is still limited data labeled in such a format. The usual approaches are based on feature engineering to correctly identify phishing campaigns, exporting lexical, syntactic, and semantic features, e.g., previous phrases. In this context, the most recent approaches have taken advantage of modern neural network architectures to record hidden information at the phrase and text levels, e.g., Long Short-Term Memory (LSTM) and Convolutional Neural Networks (CNNs). However, these models lose semantic information related to the specific problem, resulting in a variation in their performance, depending on the different data sets and the corresponding standards used for labeling. In this paper, we propose to extend word embeddings with word vectors that indicate the semantic similarity of each word with each phishing campaigns template tag. These embedded keywords are calculated based on semantic subfields corresponding to each phishing campaign tag, constructed based on the automatic extraction of keywords representing these tags. Combining general word integrations with vectors is calculated based on word similarity using a set of sequential Kalman filters, which can then power any neural architecture such as LSTM or CNN to predict each phishing campaign. Our experiments use a data indicator to evaluate our approach and achieve remarkable results that reinforce the state-of-the-art.

## 1. Introduction

Most of the sophisticated attacks in the modern age of cybercrime are based [1], among other things, on specialized phishing campaigns [2]. Usually, a phishing campaign is carried out by falsifying information in emails which can mislead the recipient and thus direct him to enter personal information on a fake website that looks identical (clone) to the corresponding legal one [3]. Clone phishing is likely the most well-known social engineering-based hacking method. Clone phishing attacks require creating a simple service or application login form to deceive the target into thinking he is signing in to a valid form to obtain his credentials. One of the most well-known instances of this assault is the bulk dissemination of messages posing as a service or social network. The mail asks the victim to click on a link that takes them to a fraudulent login form, a visual clone of the actual login page. The victim of this form of attack clicks on the link, which generally opens a false login page and requests him to input his credentials. The attacker obtains the victim's credentials and redirects him to the actual service or social network page without the victim realizing he has been hacked. This sort of attack was formerly successful for attackers who began big-scale operations to collect many credentials from irresponsible users. The effective treatment of the above specialized criminal phishing campaigns is based on the application of a classification model that can successfully predict phishing campaigns in the broader context of communication—discussion, regardless of the problem and the topic area, as well as the classification of standards capable of highlighting and generalizing the specific situation [4].

The idea that human speech contains acts of speech comes from sociolinguistic theorists [5]. The theory of interactive actions suggests that humans not only communicate real-world information through natural language expressions but also often express the underlying intended action [6]. The first step in editing the dialogue is to highlight the interactive themes and assign a functional label to the user's input to represent the communication intentions behind each expression. This first step is crucial for an automated system to generate an appropriate response. However, according to the individualization-based approach, preferences can also be based on the analysis of the entire dialogue, rather than a single expression, to find a consistent semantic representation that captures the meaning of the dialogue [7, 8].

There is a wide range of uses for interactive themes, including representations of the true meaning of verbs in dialogue theories, dialogue modules, tags for body commentary, languages for communication between automated systems, objects for analysis in dialogue systems, and elements of a rational approach. However, there is still difficulty creating a classification of interactive themes that researchers can understand and use other than the designers of this classification [9, 10]. This difficulty stems from the different interpretations assigned by researchers to the various categories of discussion topics. This kind of confusion has led some to propose standard theories that could be well identified, understood, and used in groups. In contrast, others prefer to see dialogue as secondary, within a more general idea of rational interaction, using concepts as primitive [11, 12].

Another critical issue is the recognition of themes in a dialogue between a system and an individual. Accurate recognition of topics by a dialogue system requires a well-designed language comprehension system [13, 14]. To design such a system, the syntax, i.e., the relations between the verbs and the structure of the phrases, the semantics, i.e., the reference, and the pragmatics, i.e., the analysis of the dialogues of information exchange of communication actions, must be considered. The question is how all this is used in practice to implement a phishing campaign [2, 3, 15].

Given that actions are considered transitions from situations to situations. In contrast, dialogue functions as a particular case of action, action theories proposed by artificial intelligence research generally link different sets of actions and, in particular, a collection of effects (resulting state constraints), a group of preconditions (restrictions on the initial state) and decompositions (constitute action). Based on the above definition of action, the aspects of the situation related to the possible conditions for determining the performance of the interactive issues and those that are directly affected should be identified [14, 16, 17].

To model the problem of locating phishing campaigns in English text, we propose an innovative system of using and combining word embeddings with word vectors that indicate the semantic similarity of patterns that refer to phishing campaigns. These embedded words are calculated based on semantic subfields corresponding to interactive theme tags constructed based on the automatic extraction of keywords that are representative tags that can accurately identify phishing campaigns. The architecture of the proposed system is based on successive Kalman sequential filters of continuous time to draw conclusions which can then feed a neural learning architecture, e.g., CNN [18, 19] or LSTM [20–22], to predict each phishing campaign. It should be noted that while considerable efforts have been made to model the problem of identifying phishing campaigns, a technique similar to the one proposed has not been identified in the literature.

## 2. Related Literature

This chapter discusses the current methodologies, tools, and approaches for phishing detection. Machine learning is now exhibiting its efficiency in a wide variety of applications. This technology has risen to prominence in recent years because of the rise of big data [23]. Because of big data, machine learning algorithms can now find finer-grained trends and create more exact and timely forecasts than they have ever been able to do previously [24]. Deep learning algorithms are used to identify objects in photos [25], convert spoken words to text [26], match news articles and goods to user interests, and show relevant search results [27].

Basit et al. [4] reviewed the literature on Artificial Intelligence strategies for phishing detection, including Machine, Deep and Hybrid Learning, and Scenario-based techniques. Additionally, they compared other research identifying phishing attacks using each AI technology and discussed the advantages and disadvantages of these techniques. Additionally, they offered a complete list of current phishing attack issues and future research directions on this subject.

Garces et al. [28] discussed their research on anomalous behavior related to phishing web attacks and how machine training approaches may be applied to combat the problem. A contaminated data set and scripting tools were used in this research to create machine learning models capable of identifying phishing attacks using URL analysis, which was then used in a subsequent investigation. This technique was designed to offer real-time information that may be used to make preventive choices that will mitigate the effect of an attack. Additionally, they determined that AI technology is an effective tool for dealing with this aberrant behavior since it is quicker, more efficient, and allows for the development of more advanced applications. Additionally, specific phishing strategies, such as URL shortening, may be detected by tools such as this machine learning program, which can determine if a URL is good or bad; the next step is to add the URL to a blacklist.

Bhowmic et al. [29] examined the most successful content-based email spam filtering algorithms. They concentrate mainly on Machine Learning-based junk mail and its variations and provide an overview of the related concepts, efforts, efficacy, and current state of the art. The background portion addresses the principles of email spam filtering, the evolving nature of spam, spammers' cat-and-mouse game with email service providers, and the Deep Learning front in the struggle against spam. The “Conclusion” section considers the future of email spam filtering. We conclude by evaluating the impact of Machine Learning-based filters and exploring the possible ramifications of recent technological developments in this area.

Bikov et al. [30] discussed the most prevalent attack vectors, the countermeasures necessary to limit the effect on corporate settings, and what further should be created to combat contemporary, sophisticated email assaults. None of the available anti-spam technologies can guarantee absolute efficiency against spam, phishing, or other harmful communications. It has been discovered that collecting historical email data and categorizing it by the subject property of that date and then analyzing it considerably boosts the efficacy of the supplied anti-spam system, as seen in the above analysis. It reduces the likelihood of a malicious infection or loss of organizational assets, particularly when those evaluations are carried out on an automated and frequent basis. However, the automatic execution of such procedures is substantially preferable for increased efficacy, efficiency, and resource optimization.

Mazin et al. [31] sought to examine an existing anti-spam solution and propose potential improvements. The Multi-Natural Language Anti-Spam (MNLAS) model, which is used in the spam filtering process, considers both visual information and the text of an email. The MNLAS was developed in a Java environment and can detect and filter a wide range of spam emails based on a sample of genuine emails. Anti-spam filtering systems are discovered by applying a variety of machine learning approaches, including random forest, decision tree, and support vector machine (SVM). Several limitations exist as a result of and concerning the contents and circumstances of spam email, such as the inclusion of short messages, MNL phrases, and images, among others. The vast majority of related work uses ready-made data sets that are not affected by these concerns. Visual information, short messages, and the substance of an email are all considered during the garbage filtering process by the MNLAS. The findings support the work's use in real-world circumstances. The upcoming effort will focus on validating the model against various standard data sets.

Choudhary et al. [32] demonstrated a unique strategy for detecting and filtering spam SMS messages using five machine learning classification algorithms. They examined the features of junk mail in detail and subsequently identified 10 factors that can effectively distinguish SMS spam from ham transmissions. They utilized a publicly accessible data set that was manually obtained. Their technique resulted in a high true positive rate and a false positive rate of 1.02 percent for the Random Forest classification algorithm. They intended to add more features in the future, as the best spam features assist in identifying spam messages more effectively and gathering a growing number of data sets from the real world.

### 2.1. Deep Kalman Filters

The general idea of modeling the problem follows the so-called State-Space representation and successive Kalman filters [33, 34] in estimating the maximum likelihood to identify the interactive themes that identify a phishing campaign. Specifically, the univariate mixed shape (*p*, *q*) for a stationary chronological order *Y*_*t*_ is denoted as [34]:

(1) $$\begin{array}{c} Y_{t}=\delta +\phi_{1}Y_{t-1}+\cdots +\phi_{p}Y_{t-p}+\varepsilon_{t}+\theta_{1}\varepsilon_{t-1}+\cdots +\theta_{q}\varepsilon_{t-q}. \end{array}$$

The perturbation terms *ε*_*t*_ are independent of each other, normally distributed random variables with mean zero and fluctuation *σ*^2^ white noise. Stochastic time series models of this type can be represented algebraically as state-space models by relating the *T* observations of the *y*_*t*_ series to a vector at dimension *m* *x* 1, the state vector, according to the following general equation systems [33]:

(2) $$\begin{array}{c} \begin{array}{c} y_{t}=\text{Z}\alpha_{t},\\ \alpha_{t}=\text{T}\alpha_{t-1}+\text{R}\varepsilon_{t},\varepsilon_{t}∼N\left(0,\sigma^{2}\right). \end{array} \end{array}$$

If *m* = max (*p*, *q* + 1) is set, the general form of a (*p*, *q*) model can be written as:

(3) $$\begin{array}{c} y_{t}=\phi_{1}y_{t-1}+\cdots +\phi_{m}y_{t-m}+\varepsilon_{t}+\theta_{1}\varepsilon_{t-1}+\cdots +\theta_{m-1}\varepsilon_{t-m+1}. \end{array}$$

Defining *Z*, *T*, and *R* appropriately so:

(4) $$\begin{array}{c} Z=\left(1,0,\cdots ,0\right),T=\left(\begin{array}{ccccc} \phi_{1} & 1 & 0 & \cdots & 0\\ \phi_{2} & 0 & 1 & \cdots & 0\\ \vdots & \vdots & \vdots & \ddots & \vdots \\ \phi_{m-1} & 0 & 0 & \cdots & 1\\ \phi_{m} & 0 & 0 & \cdots & 0 \end{array}\right),R=\left(\begin{array}{c} 1\\ \theta_{1}\\ \vdots \\ \theta_{m-2}\\ \theta_{m-1} \end{array}\right). \end{array}$$

Then, the linear dynamical system takes the following form, which is a state-space representation of the univariate model (*p*, *q*):

(5) $$\begin{array}{c} \begin{array}{c} y_{t}=\left(1\;0\;\cdots \;0\;\alpha_{t}\right.\\ \alpha_{t}=\left(\begin{array}{ccccc} \phi_{1} & 1 & 0 & \cdots & 0\\ \phi_{2} & 0 & 1 & \cdots & 0\\ \vdots & \vdots & \vdots & \ddots & \vdots \\ \phi_{m-1} & 0 & 0 & \cdots & 1\\ \phi_{m} & 0 & 0 & \cdots & 0 \end{array}\right)\alpha_{t-1}+\left(\begin{array}{c} 1\\ \theta_{1}\\ \vdots \\ \theta_{m-2}\\ \theta_{m-1} \end{array}\right)\varepsilon_{t} \end{array}. \end{array}$$

Once the state-space representation of the model to be estimated is found, its unknown parameters can be calculated via sequential Kalman filters [33, 34]. The Kalman filter is an iterative algorithm that allows the vector to be calculated retrospectively, given the observations *y*_1_ ⋯ *y*_*T*_. Assuming normal distributions, the condition estimator produced by the Kalman filter will be the conditionally expected value:

(6) $$\begin{array}{c} {\hat{\alpha }}_{t\;|\;s}=E\left(\alpha_{t}\;|\;y_{s},\cdots ,y_{1}\right),s<t. \end{array}$$

The Kalman filter also provides the *m* *x* *m* matrix of the condition variance-co-variance:

(7) $$\begin{array}{c} P_{t\left|s\right.}=\text{Var}\left(\alpha_{t}\;|\;y_{s},\cdots ,y_{1}\right),s<t, \end{array}$$

which serves as a measure of estimation error which is the difference between the estimated value and the true value. *P*_*t*|*s*_ is also called the mean square error matrix of ${\hat{\alpha }}_{t\left|s\right.}$.

At time *t* < *T*, the process followed is called filtering. The filter aims to update the available status vector information as the new *y*_*t*_ observation becomes available. The Kalman filter is implemented in three stages, namely, that of initialization, where the initial conditions for the state vector and its variation are set, the intermediate stage of the a priori estimation, where a pre-estimation of the state vector based on previous observations. In the final stage of the a posteriori assessment, the present observation is processed, and the appraiser resulting of the prior stage is corrected or updated afterward. When *t* > *T*, the estimator will be just the forecast for *α*_*t*_ based on the information *T*. Since, in the stationary univariable models, the error variance is constant and equal to *σ*^2^, the variance of the state vector will be set proportional to *σ*^2^, after which it is defined [35]:

(8) $$\begin{array}{c} \sigma^{2}P_{t\left|s\right.}=\sigma^{2}TP_{t-1\left|s\right.}T^{\prime }+\sigma^{2}RR^{\prime }\Rightarrow P_{t\left|s\right.}={TP}_{t-1\left|s\right.}T^{\prime }+{RR}^{\prime }, \end{array}$$

which makes it clear that the Kalman filter can be implemented independently of *σ*^2^.

Having utilized all the available information from the sample of *T* observations, the status vector has been sufficiently determined. The above results show forecasts for the value that the variable will receive for *t* periods ahead. Assuming all the parameters of the model are known, the prediction at time *t* = *T* + *l* will be the conditionally expected value and therefore using the equations of the *a priori* estimation [36, 37]:

(9) $$\begin{array}{c} \begin{array}{c} {\hat{\alpha }}_{T+\ell \left|T\right.}=T{\hat{\alpha }}_{T+\ell -1},\\ P_{T+\ell \left|T\right.}=TP_{T+\ell -1}T^{\prime }+RR^{\prime }. \end{array} \end{array}$$

In partial differential equation theory, it is also known as an a priori bound or an a priori estimate. An a priori estimate in partial differential equation theory estimates the size of a solution or the derivatives of a partial differential equation. The word a priori, which translates as “from before,” refers to the fact that an estimate for a solution is derived before it is known that a solution is possible. They are valuable for various reasons. Suppose an a priori estimate for answers to a differential equation can be demonstrated. It is usually straightforward to prove that solutions exist using the continuity approach or a fixed-point theorem.

Since the matrix *P*_*T*+*ℓ*|*T*_ is an MSE matrix, the quantity ${\hat{\alpha }}_{T+\ell \left|T\right.}$ will be an MSE prediction for the state vector.

The a posteriori estimation in the final stage of the filter is implemented so that as soon as a new observation becomes available, the status vector estimator is postupdated via the following equations [33, 38, 39]:

(10) $$\begin{array}{c} \begin{array}{c} {\hat{\alpha }}_{t}={\hat{\alpha }}_{\left.t\right|t-1}+P_{\left.t\right|t-1}Z^{\prime }\frac{v_{t}}{f_{t}},\\ P_{t}=P_{\left.t\right|t-1}-P_{\left.t\right|t-1}Z^{\prime }ZP_{\left.t\right|t-1}\frac{1}{f_{t}}. \end{array} \end{array}$$

A posteriori estimation is an estimate of an unknown variable that is equal to the posterior distribution's mode. It is similar to the probability estimation approach. Still, it uses an enhanced optimization goal that adds an estimate of the quantity to be approximated is based on a prior distribution (which quantifies the additional information available from past knowledge of a relevant event). It can be used to obtain a point estimate of an unobserved amount based on empirical data.

Respectively, the forecast will be:

(11) $$\begin{array}{c} {\hat{y}}_{T+\ell \left|T\right.}=Z{\hat{\alpha }}_{T+\ell \left|T\right.,} \end{array}$$

with a variance equal to that of the forecast error, i.e.:

(12) $$\begin{array}{c} \sigma^{2}f_{T+\ell }=\sigma^{2}ZP_{T+\ell \left|T\right.}Z^{\prime }. \end{array}$$

There are inputs and outputs to the Kalman Filter. The measurements are noisy and, at times, erroneous. The results are less noisy and, in some cases, more accurate estimations. Also, estimates of system state parameters that have not been measured or observed can be used. The overall process is shown in Figure 1.

We have seen that the state-space methodology leads through the Kalman filter to estimators with the minimum MSE and aims to determine the bound or conditional distributions of both the state vector and the sequence of *y*_*t*_ observations. In our case, the probability density function of the observation *t* will take the form [34]:

(13) $$\begin{array}{c} p\left(y_{t}\;|\;y_{t-1},\cdots ,y_{1}\right)=\frac{1}{\sqrt{2\pi \sigma^{2}f_{t}}}\exp\left(-\frac{v_{t}^{2}}{2\sigma^{2}f_{t}}\right),t=1,\cdots ,T. \end{array}$$

Consequently, the joint probability density function (PDF) will be the product of the two variables mentioned above. When the PDF is applied to a given sample (or point) in the sample space (the set of possible values for the random variable), it can be interpreted as providing a relative likelihood that the random variable's value will be close to that sample. The PDF is also known as the density of a continuous random variable. While the absolute probability for a continuous random variable to take on any particular value is zero (because there is an infinite set of possible values, to begin with), the difference between two samples of a continuous random variable can be used to infer how much more likely it is that the random variable will be close to one sample compared to the other in any given draw of the continuous random variable.

The exact probability function is factorized as follows if *y* is taken to be the total of the sample observations, and the joint probability density function is derived based on this assumption [40]:

(14) $$\begin{array}{c} L\left(\text{y}\;|\;\varphi ,\vartheta ,\sigma^{2}\right)=\overset{T}{\underset{t=1}{\prod }}\;p\left(y_{t}\;|\;y_{t-1},\cdots ,y_{1}\right)=\overset{T}{\underset{t=1}{\prod }}\;\frac{1}{\sqrt{2\pi \sigma^{2}f_{t}}}\exp\left(-\frac{1}{2\sigma^{2}}\overset{T}{\underset{t=1}{\sum }}\;\frac{v_{t}^{2}}{f_{t}}\right), \end{array}$$

which is maximized in terms of parameters (*φ*, *θ*), while the estimator of maximum likelihood of variation *σ*^2^ is:

(15) $$\begin{array}{c} {\overset{\wedge }{\sigma }}^{2}=\frac{1}{T}\overset{T}{\underset{t=1}{\sum }}\;\frac{v_{t}^{2}}{f_{t}}. \end{array}$$

If the distribution of *α*_0_ is fully determined and the mean *α*_0_ and the variance *Ρ*_0_ are known in advance, then the exact probability function of *y* is formed through the Kalman filter. This is true in the case of a single variable stationary model (*p*, *q*). This is always the case since the initial conditions for the Kalman filter are always the unrestricted mean and its variation. Given this fact, estimating maximum likelihood from the point of view of the proposed model is an easy way, as will be seen from the following example.

## 3. Phishing Campaigns Identification

Numerous statistical methods have been designed for phishing campsites to detect them. Yet, the design of a robust detector that can generalize is still one of the main concerns of the research community. The data set is used to evaluate the performance of the proposed system [41]. The provided data set includes 11430 URLs with 87 exported attributes. It is a complete set designed to benchmark machine learning-based phishing detection systems. The attributes come from three different categories; namely, 56 are extracted from the structure and syntax of the URLs [42], 24 are removed from the content of their respective pages, and 7 are exported through external service queries. The data set is balanced as it contains exactly 50% phishing and 50% legitimate URLs.

For system evaluation, the specific set will be applied to a modeling example, where assuming that [43–45]:

(16) $$\begin{array}{c} \alpha_{t}={\left(\alpha_{1,t},\alpha_{2,t},\cdots ,\alpha_{m,t}\right)}^{\prime } \end{array}$$

is the *m* *x* 1 state vector, it is now easy to represent the state-space representation as below:

(17) $$\begin{array}{c} \begin{array}{c} y_{t}=\left(1\;0\right)\alpha_{t},\\ \alpha_{t}=\left(\begin{array}{cc} 0 & 1\\ 0 & 0 \end{array}\right)\alpha_{t-1}+\left(\begin{array}{c} 1\\ \theta \end{array}\right)\varepsilon_{t}. \end{array} \end{array}$$

Therefore,

(18) $$\begin{array}{c} \left\{\begin{array}{c} \alpha_{1,t}=\alpha_{2,t-1}+\varepsilon_{t}\\ \alpha_{2,t}=\theta \varepsilon_{t} \end{array}\Rightarrow \left\{\begin{array}{c} \alpha_{1,t}=\theta \varepsilon_{t-1}+\varepsilon_{t}\\ \alpha_{2,t}=\theta \varepsilon_{t} \end{array}\right.\right.. \end{array}$$

So,

(19) $$\begin{array}{c} \begin{array}{c} \alpha_{t}=\left(\begin{array}{c} y_{t}\\ \theta \varepsilon_{t} \end{array}\right),y_{t}=\varepsilon_{t}+\theta \varepsilon_{t-1},\\ Z=\left(\begin{array}{cc} 1 & 0 \end{array}\right),T=\left(\begin{array}{cc} 0 & 1\\ 0 & 0 \end{array}\right),R=\left(\begin{array}{c} 1\\ \theta \end{array}\right). \end{array} \end{array}$$

We consider the above representation where:

(20) $$\begin{array}{c} \alpha_{t}={\left(y_{t}\theta \varepsilon_{t}\right)}^{\prime }. \end{array}$$

At time *t* = 1, the *a priori* estimate corresponds to the initialization as follows:

(21) $$\begin{array}{c} {\hat{\alpha }}_{0}={\hat{\alpha }}_{1\left|0\right.}=0\text{ and }P_{0}=P_{1\left|0\right.}=\left(\begin{array}{cc} \theta^{2}+1 & \theta \\ \theta & \theta^{2} \end{array}\right). \end{array}$$

The last relation for the matrix *Ρ*_0_ results from its detailed calculation:

(22) $$\begin{array}{c} \left(1/\sigma^{2}\right)E\left(\alpha_{t}\alpha_{t}^{\prime }\right). \end{array}$$

Therefore, the first prediction errors *ν*_1_ and *f*_1_ are:

(23) $$\begin{array}{c} v_{1}=y_{1}-Z{\hat{\alpha }}_{1\left|0\right.}=y_{1}\text{and }f_{1}=ZP_{1\left|0\right.}Z^{\prime }=\theta^{2}+1. \end{array}$$

Writing

(24) $$\begin{array}{c} P_{1\left|0\right.}=\left(\begin{array}{cc} f_{1} & \theta \\ \theta & \theta^{2} \end{array}\right) \end{array}$$

and applying the *a posteriori* equations:

(25) $$\begin{array}{c} {\hat{\alpha }}_{1}=\left(\begin{array}{c} y_{1}\\ \theta \frac{v_{1}}{f_{1}} \end{array}\right)\text{ and }P_{1}=\left(\begin{array}{cc} 0 & 0\\ 0 & \frac{\theta^{4}}{\theta^{2}+1} \end{array}\right). \end{array}$$

In the next step (*t* = 2), the *a priori* estimates will be:

(26) $$\begin{array}{c} {\hat{\alpha }}_{2\left|1\right.}=\left(\begin{array}{c} \theta \frac{v_{1}}{f_{1}}\\ 0 \end{array}\right)\text{and }P_{2\left|1\right.}=\left(\begin{array}{cc} \frac{\theta^{4}+\theta^{2}+1}{\theta^{2}+1} & \theta \\ \theta & \theta^{2} \end{array}\right), \end{array}$$

which means that:

(27) $$\begin{array}{c} v_{2}=y_{2}-\theta \frac{v_{1}}{f_{1}}\text{ and }f_{2}=\frac{\theta^{4}+\theta^{2}+1}{\theta^{2}+1}. \end{array}$$

Re-informing estimators will give:

(28) $$\begin{array}{c} {\hat{\alpha }}_{2}=\left(\begin{array}{c} y_{2}\\ \theta \frac{v_{2}}{f_{2}} \end{array}\right)\text{ and }{\text{P}}_{2}=\left(\begin{array}{cc} 0 & 0\\ 0 & \frac{\theta^{6}}{\theta^{4}+\theta^{2}+1} \end{array}\right). \end{array}$$

For *t* = 3, the *a priori* estimators will have the form:

(29) $$\begin{array}{c} {\hat{\alpha }}_{3\left|2\right.}=\left(\begin{array}{c} \theta \frac{v_{2}}{f_{2}}\\ 0 \end{array}\right)\text{and }P_{3\left|2\right.}=\left(\begin{array}{cc} \frac{\theta^{6}+\theta^{4}+\theta^{2}+1}{\theta^{4}+\theta^{2}+1} & \theta \\ \theta & \theta^{2} \end{array}\right). \end{array}$$

So,

(30) $$\begin{array}{c} v_{3}=y_{3}-\theta \frac{v_{2}}{f_{2}}\text{ and }f_{3}=\frac{\theta^{6}+\theta^{4}+\theta^{2}+1}{\theta^{4}+\theta^{2}+1}. \end{array}$$

Repeating the procedure for every *t* to *T*, it seems that the Kalman filter essentially calculates the prediction error from the retrospective equation [33, 34]:

(31) $$\begin{array}{c} v_{t}=y_{t}-\frac{\theta }{f_{t-1}}v_{t-1}, \end{array}$$

with *v*_0_ =0 and *f*_*t*_ from the relation:

(32) $$\begin{array}{c} f_{t}=\frac{\theta^{2t}+\theta^{2\left(t-1\right)}+\cdots +\theta^{2}+1}{\theta^{2\left(t-1\right)}+\cdots +\theta^{2}+1}. \end{array}$$

So, in general:

(33) $$\begin{array}{c} f_{t}=\left\{\begin{array}{c} \frac{1-\theta^{2\left(t+1\right)}}{1-\theta^{2t}},\left|\theta \right|\neq 1\\ \frac{t+1}{t},\left|\theta \right|=1 \end{array}\right.. \end{array}$$

The above is precisely the relationships we find through the modified analysis but at a lower computational cost. The dimensions of the inverted matrices have been reduced to 2 instead of *T*, which is charged as a serious advantage of the method. Replacing them also allows the probability function to be maximized numerically, using appropriate nonlinear iterative methods.

For the evaluation of the proposed system, the process results were introduced in two types of deep learning architectural networks (CNN and LSTM) with the corresponding ones of the same architecture but without the input of the results of the proposed filters [10, 21, 27, 46, 47]. The results obtained and the comparison between them is presented in Table 1.

One parameter for evaluating classification models is accuracy. Accuracy is defined as follows on a formal level: this statistic reflects how well the model performs across all classes and is used to evaluate its accuracy. It is beneficial when all of the classes are of similar significance to the student. Heuristics are used to compute this as the ratio of correct guesses to the total number of forecasts. In other words, accuracy refers to the proportion of accurate predictions provided by our model and defined as:

(34) $$\begin{array}{c} \text{Accuracy}=\frac{\text{TP}+\text{TN}}{\text{TP}+\text{TN}+\text{FP}+\text{FN}}. \end{array}$$

The precision of a model is a measure of how accurate it is in classifying a sample as positive. The following is an explanation of precision:

(35) $$\begin{array}{c} \text{Precision}=\frac{\text{TP}}{\text{TP}+\text{FP}}. \end{array}$$

The recall measures detection of positive samples by the model. There are more positive samples found when the recall is higher. As previously stated, recall is defined as:

(36) $$\begin{array}{c} \text{Recall}=\frac{\text{TP}}{\text{TP}+\text{FN}}. \end{array}$$

The following is how the *F*-score is defined:

(37) $$\begin{array}{c} F-\text{score}=\frac{\text{TP}}{\text{TP}+1/2\left(FP+FN\right)}, \end{array}$$

where TP = true positives, TN = true negatives, FP = false positives, and FN = false negatives.

The Receiver Operating Characteristic (ROC) curve depicts the performance of a classification model across all classification criteria. The above table shows the clear superiority of the method of use of the proposed filters where their use maximized the results in both cases of use of deep learning neural networks [27, 33, 48]. To be more specific, the high accuracy of the suggested model suggests that it is reliable in categorizing positive samples. In contrast, the high recall implies that the model accurately classified many positive cases. Although both positive and negative samples were identified correctly, accuracy and recall only looked at the positive issues. Therefore, while both negative and positive models impact high accuracy, high recall is only affected by positive models (and is not affected by the negative samples) according to the suggested model, consistent with previous research. The high precision considers when a selection is classified as positive, but it is indifferent to accurately categorizing all positive models in the first place. It is crucial to have high recall since it ensures that all positive examples are accurately classified, but it is unconcerned if a negative sample is mistakenly classified as positive. It successfully detects the bulk of positive data while producing many false positives compared to the other models, which have a high recall but poor accuracy (i.e., classifies many negative samples as positive). Additionally, the different models have high precision but limited recall, are correct when classifying a sample as positive but with only a small number of positive examples, and are accurate when classifying a sample as negative.

In conclusion, embedded words that are calculated based on semantic subdomains corresponding to each phishing campaign tag and constructed based on the automatic extraction of keywords that are considered representative of those tags are used as demonstrated experimentally in combining with the vectors similarity of words using a set of consecutive Kalman filters such as the one designed and analyzed above, the results of which can now power a CNN to predict each phishing campaign [4, 15, 27].

## 4. Conclusion

A highly advanced word embeddings system with word vectors that indicate the semantic similarity of each word to each phishing campaigns template tag, based on Kalman Filters, was proposed in this paper. The general idea of this process is based on the production of random but artificial data based on the theoretical probability functions of the random variables of the system under study. Therefore, firstly, it is necessary to provide statistically random numbers and create designs with the theoretical properties that we want to study. Using a sufficiently large number of iterations during random sampling and analyzing the behavior of simulated systems, it is possible to obtain a comprehensive picture of the corresponding behavior of phishing campaigns.

The advanced technique proposed where the embedded words are calculated based on semantic subspaces corresponding to each phishing campaign tag and constructed based on the automatic extraction of keywords that are considered representative in detecting dialectical parameters referred to phishing campaigns. Combining general word integrations with vectors is calculated based on word similarity using a set of sequential Kalman filters, which can then power any neural architecture such as LSTM or CNN to predict each phishing campaign.

At the assessment level, the quality of the sample sampling of the appraisers was evaluated based on the usual measures and stations, i.e., in terms of bias and MSE. At the same time, emphasis was placed on the statistical significance of the appraisers to create a picture of the confidence level of the proposed method and the performance of the estimators of each model in terms of forecasting for periods outside the sample both in terms of covering the respective confidence intervals and their accuracy concerning the theoretical samples.

The further investigation of the ways of adapting the filters to processes of modern and asynchronous change of the initial parameters of the evaluators is a critical process for the further development of the proposed model. Accordingly, the extension and empirical investigation of the properties of the method estimators in finite samples, which requires the use of Monte Carlo simulations, is also an essential evolutionary parameter of the proposed system.

## Figures and Tables

**Figure 1:** Flowchart Kalman filter. It is a real-time algorithm that can accurately estimate observable and unobservable parameters as a recursive estimator. The estimated state from the previous time step and the current measurement is required for the current state estimation. Compared to batch estimating approaches, there is no requirement for a historical record of observations and evaluations. Precision predictions are made possible by the use of high-accuracy estimations.

**Table 1:** Performance of compared methods.

Model	Accuracy	ROC	F-score	Precision	Recall
LSTM-Kalman filter	0.9986	0.9995	0.9990	0.9990	0.9989
LSTM	0.9212	0.9680	0.9215	0.9214	0.9216
CNN-Kalman filter	0.9926	0.9980	0.9925	0.9930	0.9928
CNN	0.9147	0.9670	0.9145	0.9146	0.9145

## Data Availability

Data will be provided upon request to authors.
